The article "Severe Acute Pancreatitis Rapidly Developed Into Pulmonary Edema and Diffuse Alveolar Hemorrhage Leading to Respiratory Failure: An Autopsy Case" was published in 2023. Journal: Cureus.

# Severe Acute Pancreatitis Rapidly Developed Into Pulmonary Edema and Diffuse Alveolar Hemorrhage Leading to Respiratory Failure: An Autopsy Case

**DOI:** 10.7759/cureus.46560

**Published:** 2023-10-06

**Authors:** Michiko Hosaka, Terufumi Kubo, Takeshi Matsuoka, Tadashi Hasegawa

**Affiliations:** 1 Department of Surgical Pathology, Sapporo Medical University, Sapporo, JPN; 2 Department of Pathology, Sapporo Medical University, Sapporo, JPN; 3 Department of Neurology, Date Red Cross Hospital, Date, JPN

**Keywords:** autopsy, diffuse alveolar hemorrhage, pulmonary edema, diabete mellitus, severe pancreatitis

## Abstract

Acute pancreatitis often results in life-threatening situations, making a prompt and accurate diagnosis cardinally important. To achieve these, it is crucial to correctly identify characteristic symptoms and test findings. However, when patients do not exhibit distinctive symptoms during a physician's examination, in addition to limited resources, these can become challenging. In this manuscript, we present an instructive case.

A male in his twenties, who complained of generalized malaise, was admitted to our hospital. Unfortunately, however, he passed away within two days prior to undergoing detailed examinations or receiving therapeutic interventions. We performed an autopsy in order to ascertain the reasons for this outcome. The findings revealed that pulmonary edema and diffuse alveolar hemorrhage were the causative factors of his demise, with acute pancreatitis observed in the background.

The occurrence of acute pancreatitis leading to death in youths is infrequent. Where could we have intervened to halt such an unfortunate course in a young individual? This patient probably had diabetic ketoacidosis and hyperlipidemia, both of which are known to be closely associated with acute pancreatitis. In retrospect, we should have noticed this point. In this case, the condition progressed too rapidly for appropriate therapeutic interventions. We believe that this case would provide educational instruction for similar situations that could arise in the future.

## Introduction

In this case report, we present an autopsy case of a severely obese male in his twenties with previously undetected type 2 diabetes (T2D) who had a rapid onset of acute bilateral diffuse alveolar hemorrhage and pulmonary edema, leading to respiratory failure. Acute pancreatitis was identified as the underlying cause.

Acute pancreatitis is a potentially life-threatening abdominal condition. Prompt and accurate diagnosis of acute pancreatitis is crucial for appropriate treatment [1]. Nevertheless, this presents significant challenges when patients lack apparent symptoms and there are restricted choices for tests and available healthcare personnel in a holiday hospital setting. Moreover, severe acute pancreatitis in individuals in their twenties is rare, and the mortality rate due to pancreatitis in patients in their twenties is reported to be less than one percent [2]. However, we must not forget that obesity and diabetes are risks for acute pancreatitis [3,4]. In this case, the condition progressed rapidly, preventing timely intervention. This case would provide educational instruction for similar situations that could arise in the future.

The article "Severe Acute Pancreatitis Rapidly Developed Into Pulmonary Edema and Diffuse Alveolar Hemorrhage Leading to Respiratory Failure: An Autopsy Case" was published in 2023. Journal: Cureus.

## Case presentation

A 22-year-old man with a history of hypertension had been experiencing fatigue for about a month. He had no family history of hereditary pancreatitis. Although he had visited a clinic and was confirmed negative for severe acute respiratory syndrome coronavirus 2 (SARS-CoV-2), no further detailed examination was performed. On the day of his visit, he complained of fatigue and inappetency. He visited the emergency room during the night and was admitted for observation. On admission, his body mass index was 30.8, body temperature 36.8°C, respiratory rate 16/min, pulse 101/min, blood pressure 134/72 mmHg, and SpO2 99% (room air). Although he had mild tenderness in the right hypochondrium, there was no other remarkable physical finding. Blood tests revealed elevated levels of aspartate aminotransferase (106 U/L), alanine aminotransferase (239 U/L), and lactate dehydrogenase (233 U/L), as well as an increased white blood cell count (11800 /μL) and a mild elevation of C-reactive protein. Hemoglobin and hematocrit were mildly increased to 18.1 g/dL and 52.7%, respectively, with no findings suggestive of anemia. Blood urea nitrogen level (13.2 mg/dL), creatinine level (0.78 mg/dL), and estimated glomerular filtration rate (104.9 mL/min/1.73m^2^) were all within the normal range suggesting no renal dysfunction. Plain computed tomography (CT) scan showed a fatty liver, but no pancreatitis was found (Figure 1).

**Figure 1:** Abdominal plain CT findings upon admission. The liver demonstrates lower attenuation compared to the spleen. The characteristic feature of acute pancreatitis, which is the increase in peripancreatic fat density, is not clearly observed.

Initially, his fatigue was postulated to be attributed to some form of liver damage, including hepatitis. On the day following admission, his fatigue did not improve, and he complained of right hypochondrial pain, thirst, and nausea. He was unable to consume food, yet he exhibited self-ambulation and a substantial intake of ice cream and beverages. About 28 hours post-admission, he developed acute abdominal distress. Intravenous acetaminophen was administered to the patient. Approximately 30 hours subsequent to admission (early morning), he was sleeping but opened his eyes to the nurse's prompting, stating that his abdominal pain had improved. His abdominal pain showed signs of amelioration. However, around 31 hours after admission, he was discovered to be in a state of cardiopulmonary arrest. He did not respond to resuscitation efforts and succumbed. After his death, it was revealed that his pre-mortem additional blood test had indicated an HbA1c level of 13%. We performed an autopsy with the permission of the patient’s family about six hours after his death.

The article "Severe Acute Pancreatitis Rapidly Developed Into Pulmonary Edema and Diffuse Alveolar Hemorrhage Leading to Respiratory Failure: An Autopsy Case" was published in 2023. Journal: Cureus.

Upon macroscopic examination, evident abdominal skin striations were noted on his body. Mild edema was observed in the lower legs. The oral cavity exhibited reddish liquid with bubble formation. Subepicardial serous hemorrhage was observed within the epicardium, while submucosal hemorrhage was apparent in the esophagus, duodenum, and colon. In addition, both lungs (right: 325 g, left 300 g) exhibited a deep red coloration accompanied by minimal to nearly absent air content (Figures 2A, 2B). Microscopic examination revealed widespread and intense alveolar hemorrhage and pulmonary edema across all lung lobes (Figures 2C, 2D). There was no neutrophil response to hemorrhage at either location of the lung. The heart was 470 g in weight. Histologically, myocardial tissue was preserved, with no hemorrhage, neutrophilic infiltrate, necrosis or fibrosis. There was no occlusion of the right or left coronary artery. The myocardial histology showed no lesions in the heart that could explain the pulmonary findings.

**Figure 2:** Autopsy findings of the lungs. (A, B) Macroscopic observation (after fixation with formalin): Both lungs (A: right, B: left) are firm and brownish in color, lacking aeration. Bars=1 cm. (C) Alveolar spaces are filled with fresh red blood cells, illustrating the pattern of diffuse alveolar hemorrhage. Bar=100 μm. (D) In addition to alveolar hemorrhage, pulmonary edema is observed. Bar=100 μm.

The cut surface of the pancreas demonstrated a brownish discoloration, predominantly around the main pancreatic duct (Figure 3A). Microscopically, the grossly brownish areas exhibited necrosis. Around the necrotic pancreas and adjacent adipose tissue, there was an infiltration of neutrophils that stained positive for myeloperoxidase (MPO), indicative of acute pancreatitis (Figures 3B, 3C). The pancreatic islets of Langerhans were preserved, displaying insulin-positive signals; a few CD3-positive lymphocytes were also observed, yet without eliciting isletitis (Figures 3D-3F).

**Figure 3:** Autopsy findings of the pancreas. (A) Macroscopic observation (after fixation with formalin): The cross-sectional view of the pancreas exhibited a brownish around the main pancreatic duct (arrows). Bar=1 cm (B, C) The pancreatic tissue in this region revealed extensive necrosis on histological examination, accompanied by infiltrating neutrophils that stained with (B) hematoxylin-eosin (HE) and (C) myeloperoxidase (MPO). Bars=50 μm. (D) HE staining image of pancreatic tissue. Bar=200 μm. (E) Insulin-positive cells remain in the non-necrotic pancreatic tissue. Bar=200 μm. (F) There is no infiltration of CD3-positive cells into the pancreatic tissue. Bar=200 μm.

The article "Severe Acute Pancreatitis Rapidly Developed Into Pulmonary Edema and Diffuse Alveolar Hemorrhage Leading to Respiratory Failure: An Autopsy Case" was published in 2023. Journal: Cureus.

Amyloid deposition was not discernible in the pancreatic islets of Langerhans. No adrenal tumors were identified, and adrenal enlargement was not apparent. Renal glomerular lesions were absent, and vascular abnormalities were not detected in any of the examined organs.

## Discussion

A young man in his twenties, who was obese, succumbed to respiratory failure due to sudden alveolar hemorrhage and pulmonary edema. Unfortunately, this case occurred during a holiday period with restricted diagnostic resources, and the case held insights that were solely unveiled through a postmortem pathological examination.

We postulate that acute pancreatitis was the underlying trigger for the sequence of events culminating in his demise. Although it could be challenging at the autopsy to distinguish between pancreatic necrosis and postmortem autolysis, the presence of neutrophil infiltration with positive MPO staining indicated the presence of antemortem acute pancreatitis. Our hypothesis is that he had either sudden onset or rapidly exacerbated acute pancreatitis, triggering the release of pancreatic enzymes into the bloodstream. Then he developed abrupt pulmonary edema and widespread alveolar hemorrhage. The absence of a neutrophilic response to bleeding further supports the rapid progression. The surge in vascular permeability accounts for the pulmonary edema, while the alveolar hemorrhage is attributed to disseminated intravascular coagulation (DIC) [5,6]. The occurrence of submucosal and serosal hemorrhages indicates a propensity toward systemic bleeding.

So, when did acute pancreatitis occur in this case? At the time of his admission, the patient did not exhibit the typical symptoms of pancreatitis, such as abdominal or back pain. Furthermore, CT imaging did not reveal any signs of pancreatitis. Although CT can detect early pancreatitis with a sensitivity of 60-95%, measurement of blood pancreatic enzyme, which detects pancreatitis with a sensitivity of 96.6% and specificity of 99.4%, was not performed at the admission [7,8]. The appropriateness of routine blood testing of lipase as a screening tool for acute pancreatitis in the emergency room remains unestablished [9]. Even if he had developed pancreatitis undetectable by CT upon arrival at the emergency room, according to Ranson's criteria, he did not meet any of the risk factors except for the unknown blood glucose level [10]. Based on a previous study where neutrophil infiltration was observed within 1 to 3 hours after onset in experimentally induced pancreatitis models, it is conceivable that the patient developed acute pancreatitis at severe abdominal pain that he was aware of about 3 hours before death [11]. If pancreatitis was the cause of diabetes mellitus, the histology should have shown chronic inflammatory findings corresponding to this period, since the patient had pancreatitis for at least one month, reflecting a high HbA1c level. The pancreatic tissue in this case showed predominantly neutrophilic infiltration, which we judged to be an acute phase finding.

The article "Severe Acute Pancreatitis Rapidly Developed Into Pulmonary Edema and Diffuse Alveolar Hemorrhage Leading to Respiratory Failure: An Autopsy Case" was published in 2023. Journal: Cureus.

The incidence of severe acute pancreatitis in individuals in their twenties is not high [2]. However, this patient had untreated severe diabetes mellitus in addition to severe obesity. Both obesity and diabetes are risk factors for acute pancreatitis [3,4,12]. Although a diagnosis based on laboratory data was not obtained, his excessive thirst and polydipsia could have indicated diabetic ketoacidosis (DKA). In addition, the presence of hypertriglyceridemia can be inferred from his fatty liver. Some studies have indicated the triad of DKA, hypertriglyceridemia, and acute pancreatitis, known as the “Enigmatic triangle” [13,14]. However, the definitive mechanism of how severe obesity or diabetes increases the risk of acute pancreatitis remains uncertain.

What type of diabetes was he suffering from? The prevalence of T2D as the so-called metabolic syndrome associated with insulin resistance in young Japanese individuals has been increasing [15]. Considering his age, however, autoimmune diabetes could not be ruled out. While not applicable to fulminant type 1 diabetes (T1D), if the patient had subacute-onset T1D, his elevated HbA1c levels and obesity may not contradict the diagnosis of T1D. According to the autopsy findings, T1D can be ruled out as insulin-expressing cells remained in the pancreatic tissue and isletitis due to T-cell infiltration wasn't observed. Nevertheless, determining whether his diabetes can be attributed to T2D arising from insulin resistance due to obesity in a young man is not straightforward. The possibility of endocrine disorders, including Cushing's disease and Cushing's syndrome, still remains. Although adrenal enlargement was absent, it has been reported that Cushing's disease is not always associated with adrenal enlargement [16]. Since cranial examination was not permitted, exploration of the pituitary gland could not be conducted. We did not identify any tumors capable of producing ACTH or glucagon. The distinctive red dermal striae observed externally are a characteristic finding in approximately 40% of patients with Cushing's syndrome [17]. However, since this finding can also occur in obesity other than Cushing's syndrome, it lacks diagnostic specificity. Thus, it remains inconclusive how he developed diabetes. Anyway, it can be argued that his diabetes should have been detected earlier through annual health check-ups or during previous medical visits, allowing for more timely and appropriate management. The pandemic of COVID-19 may have hindered access to healthcare, potentially resulting in the loss of these opportunities [18].

The article "Severe Acute Pancreatitis Rapidly Developed Into Pulmonary Edema and Diffuse Alveolar Hemorrhage Leading to Respiratory Failure: An Autopsy Case" was published in 2023. Journal: Cureus.

## Conclusions

Fatal cases from a sudden-onset respiratory failure consequent to such acute pancreatitis in young patients are scarcely documented. This patient's situation was exacerbated by limited medical access due to the COVID-19 pandemic and the hospital's inadequate resources at the time of onset. We present this case as an instructive example, though typical, where everything progressed in the worst possible manner.
